The article "Analysis and Prediction of Corporate Finance and Exchange Rate Correlation Based on Machine Learning Algorithms" was retracted in 2023. Reasons: signs of a paper mill; suspected computer-generated content; unreliable results or conclusions; concerns about the data.

# Analysis and Prediction of Corporate Finance and Exchange Rate Correlation Based on Machine Learning Algorithms

**DOI:** 10.1155/2022/2850604

**Published:** 2022-06-24

**Authors:** Ke Zhang, Xiaofei Wang, Junjie Wang, Sinan Wang, Feng Hui

**Affiliations:** ^1^Guosen Securities Co Ltd, Shenzhen 518000, China; ^2^Shanghai Lilith Technology Corporation, Shanghai 200030, China; ^3^Huafu Securities Co Ltd, Hangzhou 310000, China; ^4^Kaiyuan Securities Co Ltd, Xi'an 710000, China; ^5^Xigema Certified Public Accountants (Special Ordinary Partnership), Xi'an 710024, China

## Abstract

Based on the risk management of exposure to foreign exchange assets and liabilities and the application of financial derivatives, this paper provides an in-depth analysis of the financial and exchange rate risks of foreign-funded enterprises. Therefore, a method of evaluating the financial performance of listed financial enterprises based on principal component analysis and neural network model is proposed. First, principal components of alternative financial performance input-output indicators are extracted using principal component analysis. Subsequently, these principal components are used as input-output data for the DEA model to derive the relative validity evaluation results of the financial performance of individual financial enterprises and to provide a reference for decision making to improve the financial performance level of financial enterprises. Combined with the economic business data of the enterprises, an empirical test on exchange rate risk management is conducted and relevant suggestions are made on how foreign enterprises can reduce exchange rate risk losses. It has important theoretical value and practical significance for enterprise finance and exchange rate management.

## 1. Introduction

For a longer period of time in the future, it will also be difficult for the RMB to become a freely convertible currency on a global scale [1]. Moreover, on a global scale, as the world economy continues to develop, buyers dominate the trade market, which means that “in the settlement of foreign trade exports” [2]. Therefore, against the backdrop of the expected appreciation of the RMB, Chinese enterprises in a passive position are bound to face huge exchange rate risk losses [3]. As the manager of a company, whether the accountant is proficient in financial management will determine the future survival and development of foreign companies [4].

Financial accountants should be actively involved in the signing of foreign trade contracts, and the exchange rate should be taken into account to provide for a mutually acceptable risk ratio as an additional clause in the contract [5]. As foreign trade is a matter of bilateral transactions, both parties to the transaction wish to reduce the exchange rate risk, and therefore, the choice of currency of denomination is likely to be contradictory [6]. The compromise options available to both parties to foreign trade are the party with the favourable currency of denomination is required to offer other concessions to the party with the unfavourable currency; a mix of soft and hard currencies for denomination, with both parties sharing the risk; and if both parties hold mutual claims and debts, the same currency may be chosen for denomination [7]. Although Chinese foreign companies are in a passive position in the international trade market, if accountants are able to take advantage of favourable contractual terms, they will be able to reduce their exchange rate risk losses to a large extent. As the financial manager of an enterprise, the accountant must not only be proficient in financial accounting but also, and more importantly, be knowledgeable and up-to-date with the relevant knowledge of international trade contract regulations. In the negotiation of foreign trade contracts, accountants should grasp the elements of the contract terms and conditions and strive to achieve “watertightness” [8].

The article "Analysis and Prediction of Corporate Finance and Exchange Rate Correlation Based on Machine Learning Algorithms" was retracted in 2023. Reasons: signs of a paper mill; suspected computer-generated content; unreliable results or conclusions; concerns about the data.

The use of the buy-sell position balancing method does not aim to completely eliminate foreign exchange risk [9] but to minimise foreign exchange risk losses. Enterprises can achieve a certain degree of balance in their buying and selling positions by adjusting the timing of export receipts and import payments and foreign exchange loan repayments [10]. The buy-sell position balancing method is the most basic method of foreign exchange risk management, and it is also the most effective and lowest cost method; therefore, in foreign exchange risk management, enterprises should first choose this method [11]. Cross-compensation risk refers to the cross-balancing of two different foreign exchange buying and selling positions to hedge foreign exchange risk. For example, if the Hong Kong dollar is linked to the US dollar, the two currencies can be cross-balanced. Cross-balancing risk is a low-cost method of managing foreign exchange risk, whereby companies first balance their buying and selling positions in the same currency and then seek to cross-balance their buying and selling positions [12].

Whether it is a financial enterprise or an enterprise performance evaluation, related research has made some progress, but on how to establish a financial performance indicator system reflecting the financial management level of financial enterprises and how to judge the level of financial performance, these studies are still relatively few. In view of this, this paper integrates the advantages of principal component analysis and data envelopment methods in dealing with the comprehensive evaluation of multiple indicators and proposes a financial performance evaluation method based on PCA-DEA for financial enterprises. Firstly, on the basis of comparing existing studies on financial performance evaluation index systems, principal component analysis is applied to preprocess alternative input-output indicators, i.e., to distil numerous input-output indicators into a few principal components with clear practical significance. Subsequently, these principal components are used as input-output data for the DEA model to derive the relative effectiveness evaluation results of the financial performance of each financial enterprise, which provides a reference for decision making to improve the financial performance level of financial enterprises.

The article "Analysis and Prediction of Corporate Finance and Exchange Rate Correlation Based on Machine Learning Algorithms" was retracted in 2023. Reasons: signs of a paper mill; suspected computer-generated content; unreliable results or conclusions; concerns about the data.

## 2. Related Work

With the gradual acceleration of China's economic restructuring, competition in the financial sector is becoming increasingly fierce and the rapid development of financial enterprises depends to a large extent on the level of their financial performance. Therefore, an effective evaluation of the financial performance of financial enterprises can provide a basis for decision making by decision makers and stakeholders and also create new value for the system and promote its healthy development.

Financial enterprises are characterised by high risk and high debt, and if problems arise, they will have a huge impact on the overall operation of the Chinese economy, therefore, relevant research on financial enterprises has been a hot spot for scholars to focus on. The study in [13] constructed an index system and model for evaluating the symbiotic capacity of financial enterprise clusters, discussed the important factors affecting the symbiotic capacity of financial enterprise clusters; pointing out the direction for the development of financial enterprise clusters in China, the study in [14] constructing a support vector machine-based approach for the measurement of financial instruments and internal accounting control efficiency, which provides a new way for quantitative analysis and evaluation of internal accounting control efficiency of financial enterprises. In order to reduce the technological risk of Chinese financial enterprises, the study in [15] used a fuzzy comprehensive evaluation method to measure the degree of technological innovation risk of Chinese financial enterprises and obtain the risk weights of technological innovation risk provides a decision support for Chinese financial enterprises to carry out technological innovation management [16]. In order to verify whether there is a dynamic relationship between listed financial enterprises and the national macro economy, the study in [17] constructed three dynamic effect models to confirm that the effective introduction of monetary policy can play a significant role in the performance development of listed financial enterprises and provided a basis for the implementation of financial policies in China [18]. The results showed that the two were negatively correlated, and the higher the level of noninternationalisation of financial firms, the greater the negative impact of the degree of internationalisation on performance.

The article "Analysis and Prediction of Corporate Finance and Exchange Rate Correlation Based on Machine Learning Algorithms" was retracted in 2023. Reasons: signs of a paper mill; suspected computer-generated content; unreliable results or conclusions; concerns about the data.

The evaluation of financial performance, which can reflect the operation of enterprises, has been the focus of scholars' attention, and there are many relevant research results [17] that constructed a set of enterprise value evaluation index system based on the enterprise performance evaluation index system and conducted empirical research using grey clustering hair [18]. Based on the enterprise performance evaluation system promulgated by the Ministry of Finance, the hierarchical analysis method and correlation analysis method were used to evaluate the financial performance of Chinese real estate listed companies. Although these methods can achieve certain results, some evaluation models are not ideal, such as AHP, expert scoring, and other qualitative methods, and are highly subjective and cannot dynamically reflect the change pattern of financial performance data.

## 3. Corporate Financial Performance Indicator System

### 3.1. Sample Data

This paper mainly takes the listed financial enterprises in Shanghai and Shenzhen as the research sample, selects a total of 37 listed financial enterprises in the two cities, collects and collates the data of these listed financial enterprises that have passed the annual audit report in the CSMAR database in 2015, and selects the relevant data of the publicly disclosed financial indicators in the financial statements.

### 3.2. Selection of Indicators

This paper takes financial enterprises as the research subject, and the Ministry of Finance promulgated the measures for evaluating the performance of financial enterprises in 2016, which stipulates that the four dimensions of profitability, operating growth, asset quality, and solvency are required in evaluating the performance of financial enterprises. Therefore, based on these four dimensions and drawing on the financial indicator system constructed in the literature [18], this paper selects 26 common indicators that can measure the financial performance of listed financial enterprises at multiple levels and from multiple perspectives.

The article "Analysis and Prediction of Corporate Finance and Exchange Rate Correlation Based on Machine Learning Algorithms" was retracted in 2023. Reasons: signs of a paper mill; suspected computer-generated content; unreliable results or conclusions; concerns about the data.

Due to the large number of financial indicators and the correlation between them, it is necessary to select the indicators that can best reflect the performance from many indicators. At the present stage, the most commonly used methods for selecting financial performance indicators are the expert consultation method and the hierarchical analysis method, but the evaluation results of these two methods are affected by the structure and number of experts and are highly subjective. Therefore, based on the existing research, this paper uses solvency and asset quality as input indicators and operational growth and profitability as output indicators. In particular, solvency reflects the level of debt burden, the ability to repay various debts and the debt risk faced by financial enterprises; asset quality reflects the efficiency of financial enterprises in utilising their operating assets, asset safety, and management level; operational growth reflects the level of operational growth and capital preservation and appreciation of financial enterprises; profitability reflects the quality of profitability and the level of input and output of financial enterprises within a certain period of time. The specific indicators are shown in Table 1.

The abovementioned indicator system evaluates the financial performance of financial enterprises from several aspects. Although it satisfies the principles of scientificity and diversity in establishing an indicator system, it does not meet the principles of streamlining and feasibility, especially the rules of DEA for input-output indicators.

To solve these problems, the following will use principal component analysis to perform dimensionality reduction in order to reduce the number of dimensions of these financial performance input and output indicators and to find from them the uncorrelated principal components that reflect the main information and subsequently use the values of the principal components as the original input-output variables for DEA model analysis.

### 3.3. PCA Treatment of Alternative Input Indicators

A factor analysis of the alternative input indicators gives a KMO value of 0.574 (greater than 0.5) and a chi-square statistic significance level of 0.000 after Bartlett's test, which implies that there are common factors among the input indicators and that they are suitable for factor analysis. In terms of the amount of variance explained, the cumulative variance contribution of the five main components FAC1, FAC2, FAC3, FAC4, and FAC5 selected in the paper was 78.231%. Factor rotation was then performed using the variance maximisation method, and the results are shown in Table 2.

The article "Analysis and Prediction of Corporate Finance and Exchange Rate Correlation Based on Machine Learning Algorithms" was retracted in 2023. Reasons: signs of a paper mill; suspected computer-generated content; unreliable results or conclusions; concerns about the data.

As can be seen from the factor loading matrix, the principal component FAC1 mainly contains information on two indicators, namely, accounts receivable to revenue ratio and accounts receivable to turnover days, reflecting the efficiency of capital recovery of financial enterprises; the principal component FAC2 mainly contains information on four indicators, namely, gearing ratio, net cash flow from operating activities/liabilities, operating debt ratio, and total asset turnover ratio, reflecting the level of indebtedness, riskiness, and ability to repay principal and interest on debt of financial enterprises; the principal component FAC3 mainly contains information on three indicators, namely, long-term capital indebtedness ratio, financial debt ratio, and return on investment, reflecting the long-term capital structure of financial enterprises and their ability to absorb savings; the principal component FAC4 mainly contains information on four indicators, namely, cash assets ratio, fixed assets ratio, consolidated leverage, and return on long-term capital, reflecting the liquidity of financial enterprises, the efficiency of asset utilisation, the impact of changes in sales volume on earnings per share, and the ability of capital profitability; the principal component FAC5 contains information on two indicators, namely, equity multiplier and accounts receivable turnover ratio, reflecting the ability of financial enterprises to achieve financial leverage and liquidity turnover speed.

### 3.4. PCA Treatment of Alternative Output Indicators

Similarly, a factor analysis of the alternative output indicators gives a KMO value of 0.573 (greater than 0.5) and a chi-square statistic significance level of 0.000 after Bartlett's test, which implies that there are common factors among the output indicators that are suitable for factor analysis. In terms of the amount of variance explained, the cumulative variance contribution of the four principal components FAC1, FAC2, FAC3, and FAC4 selected in the paper was 88.354%. Subsequently, the factor rotation was performed using the variance maximisation method, and the results are shown in Table 3.

As can be seen from the factor loading matrix, the principal component FAC1 contains information on five indicators, namely, the growth rate of total assets, the growth rate of net profit, the growth rate of comprehensive income, the net operating margin, and the growth rate of return on net assets, reflecting the growth scale of financial enterprises' assets, operating results, operating income to generate net profit, and profitability and growth capacity;the principal component FAC2 contains information on three indicators, namely, capital preservation and appreciation rate, return on assets (ROA), and net profit margin on total assets , reflecting the operational efficiency and safety of financial enterprises' capital, the efficiency of asset utilisation, and profitability; FAC3 contains the relevant total operating utilization ratio, which reflects the use of human resources in the financial sector; the principal component FAC4 contains information on the total operating cost ratio, which reflects the overall situation of the financial sector and the position of the financial enterprise in the industry, and provides a comprehensive understanding of the financial situation of the enterprise.

The article "Analysis and Prediction of Corporate Finance and Exchange Rate Correlation Based on Machine Learning Algorithms" was retracted in 2023. Reasons: signs of a paper mill; suspected computer-generated content; unreliable results or conclusions; concerns about the data.

## 4. Predictive Modelling Based on Deep Belief Networks

### 4.1. Deep Belief Network Model

As an efficient deep learning algorithm, deep belief networks have gradually developed into a mainstream technological direction. A random neural network Boltzmann machine model based on statistical principles was generated, containing an implicit layer and a visible layer, as shown in Figure 1.

On these basis, the principle framework of the restricted Boltzmann machine is proposed, as shown in Figure 2.

Where *a*=(*a*_1_, *a*_2_, ⋯,*a*_*n*_*v*__)^T^ ∈ R^*n*_*v*_^ denotes the bias vector of the visible layer, *b*=(*b*_1_, *b*_2_, ⋯,*b*_*n*_*h*__)^T^ ∈ R^*n*_*h*_^ denotes the bias vector of the hidden layer and *W* = (*w*_*i*,*j*_) ∈ R^*n*_*h*_×*n*_*v*_^ denotes the weight matrix between the hidden and visible layers.

The restricted Boltzmann machine introduces a series of related probability distribution functions through the energy function. For a given set of neurons the state vector (*v*, *h*) is represented by an energy function, as in

(1) $$\begin{array}{c} E\left(v,h\;|\;\theta \right)=-\sum_{i=1}^{n_{v}}a_{i}v_{i}-\sum_{j=1}^{n_{h}}b_{j}h_{j}-\sum_{i=1}^{n_{v}}\sum_{j=1}^{n_{h}}h_{j}w_{i,j}v_{i}, \end{array}$$

where *v* denotes the state vector of neurons in the visible layer, *h* denotes the state vector of neurons in the hidden layer, *n*_*v*_ denotes the total number of all neurons in the visible layer, *n*_*h*_ denotes the total number of all neurons in the hidden layer, and *θ*={*a*_*i*_, *b*_*j*_, *w*_*i*,*j*_} denotes the conditioning factor limiting the Boltzmann machine architecture.

With the energy function defined in equation (1) , the joint probability distribution of the state (*v*, *h*) can be obtained as in

(2) $$\begin{array}{c} P\left(v,h|\theta \right)=\frac{1}{Z\left(\theta \right)}{\text{e}}^{-E\left(v,h|\theta \right)}, \end{array}$$

where *Z*(*θ*) expressions, as in

(3) $$\begin{array}{c} Z\left(\theta \right)=\sum_{v,h}e^{-E\left(v,h|\theta \right)}, \end{array}$$

where *Z*(*θ*) denotes the normalisation parameter. Let *P*(*v*|*θ*) be the probability distribution of the visible layer vector *v*. This can be calculated by *p*(*v*, *h*|*θ*) the edge distribution for *P*(*v*|*θ*), as in

(4) $$\begin{array}{c} PP\left(v|\theta \right)=\sum_{h}P\left(v,h|\theta \right)=\frac{1}{Z\left(\theta \right)}\sum_{h}e^{-E\left(v,h|\theta \right)}. \end{array}$$

In the same way, we can obtain the probability distribution of the hidden layer vector *hP*(*h|θ*) as in

(5) $$\begin{array}{c} P\left(h|\theta \right)=\sum_{v}P\left(v,h|\theta \right)=\frac{1}{Z\left(\theta \right)}\sum_{v}e^{-E\left(v,h|\theta \right)}. \end{array}$$

By analysing equations (4) and (5), it can be seen that in order to obtain *P*(*v|θ*) and *P*(*h|θ*), the key step is to calculate the normalisation parameter *Z*(*θ*). However, equation (5) shows that its computational complexity is high. However, due to the special principle that restricts the Boltzmann machine model (the visible and hidden layers are conditionally independent), the probability of a neural unit being activated in the hidden layer can be calculated by equation (6) when the states of all neurons in the visible layer are known.

(6) $$\begin{array}{c} P\left(h_{j}=1|v,\theta \right)=\sigma \left(b_{j}+\sum_{i}v_{i}w_{ij}\right), \end{array}$$

where *σ*(−) denotes the sigmoid activation function.

The article "Analysis and Prediction of Corporate Finance and Exchange Rate Correlation Based on Machine Learning Algorithms" was retracted in 2023. Reasons: signs of a paper mill; suspected computer-generated content; unreliable results or conclusions; concerns about the data.

Because all neural nodes within the same layer are connectionless with each other, the relationship between the values taken by all neural nodes within the same layer and the values taken by a single node is as in

(7) $$\begin{array}{c} P\left|\left(h|v\right)\right|=\prod_{j-1}^{n_{h}}P\left(h_{j}|v\right), \end{array}$$

(8) $$\begin{array}{c} P\left(v|h\right)=\prod_{i-1}^{n_{v}}P\left(v_{i}|h\right). \end{array}$$

A randomized gradient algorithm is usually used to find the maximum value of ∑_*i*=1_^*i*^log  *P*(*v*^(*i*)^|*θ*) in order to obtain the optimal conditioning factor *θ* in the network. A deep belief network model is used, as shown in Figure 3.

### 4.2. Deep Belief Network Training Process

The deep belief network training process is generally divided into 2 steps: a pretraining phase and a fine-tuning phase.

The loss function required for ageing in the fine-tuning phase is given in

(9) $$\begin{array}{c} L\left(x,y\right)={\left\|x-y\right\|}_{2}^{2}, \end{array}$$

where the symbol ‖.‖_2_ denotes the 2-parameter reconstruction error, *x* denotes the input data, and *y* denotes the reconstructed data.

## 5. Corporate Financial Performance Evaluation Model

When the number of evaluation indicators increases to a certain level, it will not only increase the workload of the DEA model in data processing but also make the evaluation results meaningless due to the strong interrelationship between input and output indicators causing the validity of all decision units to be close. Therefore, in order to avoid the above problems, this paper proposes a combined evaluation model based on factor analysis and DEA to evaluate the financial performance of financial enterprises [21, 22].

The article "Analysis and Prediction of Corporate Finance and Exchange Rate Correlation Based on Machine Learning Algorithms" was retracted in 2023. Reasons: signs of a paper mill; suspected computer-generated content; unreliable results or conclusions; concerns about the data.

Using the advantages of the PCA method in extracting the characteristics of indicators, the input and output data required by the DEA model are preprocessed, i.e., multiple indicators are synthesised into a few principal components that can cover their main information, in order to achieve the purpose of dimensionality reduction of the indicators [23].

The processed input and output indicators are fed into the DEA model in order to calculate the relative efficiency of the financial performance of financial enterprises. This not only retains the complete information of each indicator but also reduces the degree of correlation between indicators, while satisfying the requirements of the DEA model, so that the model can adequately evaluate the relative effectiveness of the decision-making unit and ensure the accuracy and scientificity of the results. The process is shown in Figure 4.

## 6. Evaluating Model Validity Tests

As some of the principal components obtained above have negative values, they do not meet the DEA model's requirement of positive values for the input and output variables. Therefore, the principal components obtained in the above section were normalised to obtain new input and output data, which were fed into the DEA model to obtain the results, as shown in Table 4.

Technical efficiency can measure an enterprise's ability to allocate resources and its ability to use resources efficiently in many ways and evaluate whether its industrial structure is in line with the overall requirements to enable the enterprise to maximise its economic efficiency. On the whole, these 37 listed financial enterprises operate well in terms of input-output efficiency in terms of financial performance, with an average value of 0.883 for technical efficiency, indicating that these listed financial enterprises have good capabilities in terms of capital allocation and efficiency of use.

As can be seen from Table 4, there are 24 financial enterprises with all three efficiency values of 1, accounting for 64.9% of the total sample, which are on the DEA efficiency frontier, indicating that these 24 financial enterprises are relatively efficient, achieving “maximum output with existing inputs” and “minimum input on top of existing output.” The remaining 13 financial enterprises have achieved the best efficiency in terms of capital allocation and utilisation, with no waste of input resources and no shortfall in output. The technical efficiency of the remaining 13 financial firms ranged from 0.2 to 0.9, accounting for 35.1% of the total sample, indicating that the DEA of these financial firms was ineffective, with the dual problems of inefficient capital allocation and low capital efficiency. There are two main reasons for this: firstly, technical efficiency is 1 and scale efficiency is ineffective. For example, DUM19 technical efficiency is 0.452, technical efficiency is 1, and scale efficiency is 0.452. If we want to make this firm DEA effective, we need to increase the scale of investment and adjust to scale, and we can achieve relative optimality after increasing scale efficiency. Second, neither pure technical efficiency nor scale efficiency is 1, but both are at the stage of increasing returns to scale, indicating that it is advantageous for these financial firms to expand their scale at this stage. For example, the technical efficiency of DUM2 is 0.433, the technical efficiency is 0.448, and the scale efficiency is 0.967, which are in the stage of increasing returns to scale. If you want to make this enterprise reach DEA effective, you can adjust the scale of investment to improve the technical efficiency, but you cannot ignore the improvement in technology, and you need to make comparative improvements in both financial efficiency and input scale of the enterprise in order to reach relative optimization [24].

The article "Analysis and Prediction of Corporate Finance and Exchange Rate Correlation Based on Machine Learning Algorithms" was retracted in 2023. Reasons: signs of a paper mill; suspected computer-generated content; unreliable results or conclusions; concerns about the data.

In terms of the value of pure technical efficiency, its overall sample mean reached 0.954 and the pure technical efficiency of the sample was 30 , accounting for 81% of the total sample. For the remaining seven financial enterprises with ineffective DEA, they need to upgrade their technology and increase the scale of inputs in order to achieve relative optimality. For example, DUM2 with a pure technical efficiency of 0.448 and a scale efficiency of 0.967 has a low financial efficiency mainly due to a low level of financial management and technical inputs. Therefore, for these financial companies with relatively low values of pure technical efficiency, the management should further improve the scientific nature of their operational and investment decisions and focus on managing the returns and risks of their investment projects [25, 26].

There are three types of returns to scale: constant returns to scale, diminishing returns to scale, and increasing returns to scale. Production with constant returns to scale is generally the most efficient. Increasing returns to scale indicate that each additional unit of resource input produces greater than one unit of output, while the opposite is true for decreasing returns to scale. In terms of scale efficiency coming to a value, the sample mean is 0.918, which indicates that only 0.82% of resources are underutilised at scale.

The article "Analysis and Prediction of Corporate Finance and Exchange Rate Correlation Based on Machine Learning Algorithms" was retracted in 2023. Reasons: signs of a paper mill; suspected computer-generated content; unreliable results or conclusions; concerns about the data.

In terms of returns to scale, all financial firms are at the stage of constant or increasing returns to scale, indicating the huge potential and prospects for the development of the financial sector, when financial firms continue to increase their capital investment, which can lead to increasing output, thus contributing to the rapid development of the financial system as a whole. Twenty-four financial firms have an efficiency of scale value of 1. They are in a state of constant returns to scale, and their use of resources and scale of inputs are optimal and do not need to be improved. The remaining 13 financial firms, all of which have an efficiency of scale value less than 1, are in a state of increasing returns to scale despite their inefficient scale. For these financial firms, their pure technical efficiency and scale efficiency are inefficient, and in order to reach optimality, improvements must be made in both the input and output efficiency of financial resources.

For the purpose of analysis, assume that a foreign-owned company, Company A, has the following economic operations:

1. On 4 January 2010, Company A enters into a trade contract with a foreign importer, Company B, which provides that over the next 12 months, with the 15th of each month being the shipment date, Company A will export to Company B goods valued at CNY72 million in 12 batches, with each batch being settled 60 days after the shipment date in the amount of CNY6 million.
2. On 5 January 2010, Company A launched a new domestic production line with a total project investment of CNY60 million, with an expected useful life of five years and a 30% increase in productivity, payable in 12 monthly instalments of CNY5 million from March 2010.
3. On 15 April 2010, Company A borrowed funds of CNY80 million from the Industrial and Commercial Bank of China to resolve its liquidity difficulties. Company A's foreign exchange exposure risk data (as shown in Table 5).

In the example above, the accountant did not apply any exchange rate risk management measures, and against the backdrop of a significant appreciation of the RMB, Company A, a foreign-owned company, suffered significant exchange rate risk losses. However, if the accountant had been able to use flexible foreign exchange exposure management, Company A's situation would have been different, as the price index CPI in China has been increasing since the second half of 2010 and the central bank has adopted a tightening monetary policy, which means that the cost of financing for companies will increase. In contrast, due to the low economic boom in the United States, the Federal Reserve has adopted a quantitative easing monetary policy with lower lending rates in US dollars.

The article "Analysis and Prediction of Corporate Finance and Exchange Rate Correlation Based on Machine Learning Algorithms" was retracted in 2023. Reasons: signs of a paper mill; suspected computer-generated content; unreliable results or conclusions; concerns about the data.

Therefore, Company A should choose a loan in US dollars to introduce advanced production lines from abroad and increase the rate of return of its project investment.

## 7. Conclusions

The rapid development of an enterprise depends largely on the level of its financial performance. An effective evaluation of its financial performance can create new value for the financial system continuously and promote the healthy development of the financial industry. This paper uses principal component analysis methods and data envelopment methods to conduct a comprehensive evaluation of the financial performance of the listed financial enterprises. While ensuring that the information on the indicators is retained intact, it can also provide a scientific and effective evaluation of the financial performance of financial enterprises and provide financial enterprises with the opportunity to make appropriate adjustments to their own resources or scale in order to achieve the optimal allocation of resources, thereby achieving an improvement in the overall financial performance level of financial enterprises.

## Figures and Tables

**Figure 1:** Boltzmann machine model.

**Figure 2:** Restricted Boltzmann machine model.

**Figure 3:** Depth generation model.

**Figure 4:** Financial performance evaluation process of the financial companies based on PCA and DEA.

**Table 1:** Financial performance evaluation indicator system for financial enterprises.

Input index	Name	Symbol	Output indicators	Name	Symbol
Solvency	Asset liability ratio	X1	Business growth	Rate of capital accumulation	Y1
		X2		Growth rate of total assets	Y2
	Net cash flow from operating activities/liabilities	X3		Net profit growth rate	Y3
	Operating debt ratio	X4		Growth rate of comprehensive income	Y4
	Financial liability ratio	X5		Sustainable growth rate	Y5
	Equity multiplier	X6	Profitability	Return on assets	Y6

Asset quality	Cash asset ratio	X7		Profit margin on total assets (ROA)	Y7
	Fixed assets ratio	X8		Return on net assets	Y8
	Integrated lever	X9		Operating net interest rate	Y9
	Ratio of accounts receivable to income	X10		Total operating cost rate	Y10
	Days sales outstanding	X11		Return on net assets growth rate	Y11
	Total asset turnover	X12			
	Long term return on capital	X13			
	Return on investment	X14			
	Accounts receivable turnover	X15			

The article "Analysis and Prediction of Corporate Finance and Exchange Rate Correlation Based on Machine Learning Algorithms" was retracted in 2023. Reasons: signs of a paper mill; suspected computer-generated content; unreliable results or conclusions; concerns about the data.

**Table 2:** Factor loading matrix for input indicators after orthogonal rotation.

Input indicators	Component				
	FAC1	FAC2	FAC3	FAC4	FAC5
Asset liability ratio	0.224	−0.741	−0.417	−0.174	−0.111
Long term capital liability ratio	0.049	0.075	0.974	−0.017	0.014
Net cash flow from operating activities/liabilities	−0.214	0.551	−0.044	0.357	0.471
Operating debt ratio	0.157	0.921	0.063	−0.17	−0.037
Financial liability ratio	−0.042	0.047	0.978	−0.067	0.054
Equity multiplier	0.197	−0.154	−0.287	0.247	−0.700
Cash asset ratio	−0.557	0.084	−0.063	0.714	0.247
Fixed assets ratio	−0.039	0.165	−0.224	−0.778	0.247
Integrated lever	0.178	−0.367	0.318	−0.687	−0.113
Ratio of accounts receivable to income	0.947	−0.196	−0.182	−0.047	−0.032
Days sales outstanding	0.924	−0.0203	−0.195	−0.062	−0.047
Total asset turnover	−0.387	0.789	−0.082	0.058	0.035
Long term return on capital	−0.437	−0.051	−0.247	0.662	0.017
Return on investment	−0.388	−0.043	−0.097	0.150	−0.208
Accounts receivable turnover	0.245	−0.056	−0.112	0.178	0.768

**Table 3:** Factor loading matrix for output indicators after orthogonal rotation.

Input indicators	Component			
	FAC1	FAC2	FAC3	FAC4
Rate of capital accumulation	0.074	0.861	0.235	−0.167
Growth rate of total assets	0.793	0.247	0.387	−0.094
Net profit growth rate	0.748	0.557	0.192	0.167
Growth rate of comprehensive income	0.857	−0.025	0.338	−0.036
Sustainable growth rate	0.339	0.154	0.871	0.033
Return on assets	0.196	0.952	0.146	−0.070
Total assets net profit margin (ROA)	0.193	0.951	0.157	−0.065
Return on net assets	0.062	0.472	0.834	−0.176
Total operating cost rate	0.038	−0.154	−0.095	0.939
Return on net assets growth rate	0.847	0.080	0.081	0.345

**Table 4:** Results of the 2015 financial performance evaluation of the listed financial companies.

DMU	Technical efficiency	Pure technical efficiency	Scale efficiency	Returns to scale
1	1	1	1	Unchanged
2	0.434	0.449	0.968	Increasing
3	1	1	1	Unchanged
4	1	1	1	Unchanged
5	0.643	0.747	0.847	Increasing
6	0.936	1	0.924	Increasing
7	1	1	1	Unchanged
8	1	1	1	Unchanged
9	1	1	1	Unchanged
10	1	1	1	Unchanged
11	0.727	1	0.728	Increasing
12	1	1	1	Unchanged
13	1	1	1	Unchanged
14	0.877	0.987	0.887	Increasing
15	0.651	0.874	0.744	Increasing
16	1	1	1	Unchanged
17	1	1	1	Unchanged
18	1	1	1	Unchanged
19	0.452	0.879	0.749	Increasing
20	0.231	0.438	0.527	Increasing
21	0.958	1	0.987	Increasing
22	1	1	1	Unchanged
23	1	1	1	Unchanged
24	1	1	1	Unchanged
25	0.857	1	0.858	Increasing
26	1	1	1	Unchanged
27	1	1	1	Unchanged

**Table 5:** Exposure data for Company A's foreign exchange exposure positions.

Date	Foreign exchange assets	Foreign exchange liabilities	Exchange rate	Open mouth
2010.01.15	USD6000000	2	6.8271	USD6000000
2010.02.15	USD6000000	1	6.8271	USD6000000
2010.03.15	USD6000000	2	6.8271	USD6000000
2010.04.15	USD6000000	2	6.8271	USD6000000
2010.05.15	USD6000000	5	6.8702	USD6000000
2010.06.15	USD6000000	4	6.8243	USD6000000
2010.07.15	USD6000000	4	6.7744	USD6000000
2010.08.15	USD6000000	6	6.8741	USD6000000
2010.09.15	USD6000000	6	6.5742	USD6000000
2010.10.15	USD6000000	5	6.4571	USD6000000
2010.11.15	USD6000000	6	6.5787	USD6000000
2010.12.15	USD6000000	8	6.5654	USD6000000

The article "Analysis and Prediction of Corporate Finance and Exchange Rate Correlation Based on Machine Learning Algorithms" was retracted in 2023. Reasons: signs of a paper mill; suspected computer-generated content; unreliable results or conclusions; concerns about the data.

## Data Availability

The experimental data used to support the findings of this study are available from the corresponding author upon request.
